# Cardiac Rehabilitation Improves Long-Term Prognosis for People with Chronic Kidney Disease Undergoing Percutaneous Coronary Intervention: A Propensity Matching Analysis

This article has been retracted.

**DOI:** 10.1155/2022/1196682

**Published:** 2022-02-09

**Authors:** Hong Mei Qin, Dan Zheng, Jie Wu

**Affiliations:** ^1^Department of Physical Examination Department, First People's Hospital of Chongqing Liangjiang New Area, Chongqing, China; ^2^Department of Emergency Department, First People's Hospital of Chongqing Liangjiang New Area, Chongqing, China

## Abstract

**Objectives:**

According to researches, many people with chronic kidney disease (CKD) had the higher incidence rate and mortality rate of coronary artery disease (CAD) after percutaneous coronary intervention than those who did not receive percutaneous coronary intervention, while coronary rehabilitation was beneficial for patients who received percutaneous coronary intervention I. This study aims to analyze whether coronary rehabilitation was beneficial to patients with CKD after percutaneous coronary intervention. *Patients and Methods*. A retrospective survey was used to collect clinical data of patients undergoing percutaneous coronary intervention due to CAD, and CKD patients were screened for further analysis. According to whether patients had received coronary rehabilitation treatment, research subjects were divided into two groups, the coronary rehabilitation group and the noncoronary rehabilitation group. The baseline characteristics of the propensity score matching between the two groups were compared. Survival analysis used the Cox hazard ratio (HR) model as regression method to compare the relative risk of the endpoints in the coronary rehabilitation group and the noncoronary rehabilitation group.

**Results:**

From January 2007 to January 2012, a total of 246 CKD patients treated with percutaneous coronary intervention were included in this study, and 106 of them obtained coronary rehabilitation after surgery. After propensity score matching, there were 89 pairs of patients in the two groups who had no significant difference in demographic and clinical characteristics (all *P* > 0.05). CKD patients receiving coronary rehabilitation had a significant reduction in all-cause mortality (HR 0.465, 95% CI 0.233–0.926, *P*=0.029) and cardiac complications (HR 0.532, 95% CI 0.287–0.984, *P*=0.044). Survival analysis showed that the survival rate of the coronary rehabilitation group was significantly higher than that of the noncoronary rehabilitation group (*P*=0.024).

**Conclusions:**

For CKD patients undergoing percutaneous coronary intervention, receiving cardiac rehabilitation can significantly improve long-term survival and reduce cardiac events.

## 1. Introduction

Although the mortality rate of people suffering from coronary artery disease (CAD) has been on a downward trend due to the successful development of more and more effective interventional technologies and cardiovascular drugs [1–3], serious cardiogenic death and recurrence risks still pose a serious threat to CAD patients. CAD patients are necessary for comprehensive treatment. Cardiac rehabilitation including health education level, recommendations for reducing cardiovascular accidents, physical exercise, and stress management are some of the comprehensive measures for patients with heart disease [4]. And well-designed coronary rehabilitation includes the following factors: medical assessment, prescribed exercise, correction of cardiac risk factors, education and counseling, and long-term continuous implementation [5–7]. The survey shows that although the cost of coronary rehabilitation is low and the curative effect is good, the participation rate of CAD patients is only 20% to 40% [8]. In China, the participation rate of CAD patients for coronary rehabilitation becomes worse due to the relatively undeveloped socio-economic conditions, which requires more clinical practice to promote the efficacy of coronary rehabilitation for CAD patients [9].

Chronic kidney disease (CKD) complication of CAD has attracted social attention for the increasing incidence of CAD and the long-term risks of cardiac events [10, 11]. More and more studies strongly recommend that people with acute coronary syndrome (ACS) (including ST segment elevation myocardial infarction and non-ST segment elevation myocardial infarction), with unstable angina pectoris and with undergoing reperfusion, receive coronary rehabilitation treatment [12]. In view of the current lack of relevant research data on whether coronary rehabilitation has a significant effect on ACS patients with CKD, in this study, we used a retrospective propensity matching study to analyze the prognostic intervention of long-term standardized coronary rehabilitation in people who have undergone percutaneous coronary intervention. This study provided more evidence for the benefits and indications of coronary rehabilitation.

## 2. Patients and Methods

### 2.1. Study Population

We retrospectively compiled the clinical data of patients who meet the following criteria: (1) the patient diagnosed with ACS and receiving percutaneous coronary intervention treatment according to the 2011 ACCF/AHA/SCAI guideline [13]; (2) the patient who had a history of CKD or eGFR lower than 60 mL/min/1.73 m^2^; (3) the patient who had no contraindications of coronary rehabilitation including unstable angina, severe heart failure (with LVEF < 30%), and uncontrolled ventricular arrhythmia [14]; (4) the patient who completed routine follow-up; (5) the patient who signed an informed consent of admission.

The study compared demographical characteristics, examination results during hospitalization, and long-term subsequent prognosis outcomes. The study was also approved by the hospital Medical Ethics Committee.

Accorded to the abovementioned criteria, there were 246 eligible CKD patients receiving percutaneous coronary intervention in the hospital between January 2007 and January 2012. Accorded to whether the patients had received coronary rehabilitation treatment, the research subjects were divided into two groups, the coronary rehabilitation group and the noncoronary rehabilitation group.

### 2.2. Cardiac Rehabilitation

According to the BACPR Standard 2^15^, the coronary rehabilitation program was launched in the Department of Cardiology Hospital, since February 2010, when a group of coronary rehabilitation was founded including cardiologists, nurse specialists, physiotherapists, dietitians, psychologists, exercise specialists, occupational therapists, and clerical administrators. A well-designed coronary rehabilitation plan was made for each patient who was willing to receive treatment. The coronary rehabilitation plan included the following steps: first of all, health education and habit correction; secondly, lifestyle analysis and risk factor control (outdoor activities, exercise, diet correction, and smoking cessation); third, psychological counseling and evaluation; fourth, medical evaluation and risk factor control; fifth, cardioprotective therapies; sixth, long-term follow-up on time; and seventh, regularly evaluate the coronary rehabilitation program. The patients who received coronary rehabilitation plan needed to attend the coronary rehabilitation sessions within 3 months after percutaneous coronary intervention and the multidisciplinary program must last more than 1 year (more than 3 sessions of coronary rehabilitation).

### 2.3. Follow-Up and Endpoints

The follow-up lasts from January 2010 to January 2017 by telephone or out-patient clinics; each patient was given an annual inquiry of their conditions. The data were regarded as meaningless if the patient's clinical data were incomplete or the contact was interrupted during long-term follow-up. Primary and secondary endpoint studies were as follows: the primary endpoint was defined as all-cause mortality during long-term follow-up; the secondary endpoints were defined as composite adverse outcomes, including adverse outcomes such as myocardial infarction and unexpected revascularization and so on.

### 2.4. Statistical Analysis

In this study, IBM SPSS Statistics version 19.0 (SPSS, Inc, Armonk, NY) was used for statistical analysis. Firstly, the normal distribution test of variables was carried out to check the distribution of variables. Continuous variables conforming to normal distribution were expressed as mean ± standard deviation, and classified variables were expressed as proportion.

The comparison of continuous variables between the two groups used the independent sample *t*-test. The chi-square test was performed in different evaluations of categorical variables. Multiple logistic regression was performed to calculate propensity scores by considering demographic and clinical variables. Use the “greedy matching” method to match patients with the closest propensity score. After propensity score matching, Student's *t*-test and McNemar paired sample were used for analysis.

Survival analysis used Cox hazard ratio (HR) model as a regression method to compare the relative risk of the endpoints in the coronary rehabilitation group and the noncoronary rehabilitation group. We performed univariate analysis between covariates and endpoints. The Kaplan–Meier survival curve and log rank test were used to compare the survival status of the coronary rehabilitation group and the noncoronary rehabilitation group. *P* value less than 0.05 was considered as statistically significance.

## 3. Results

### 3.1. Patient Characteristics

There were 246 eligible research subjects that were included in this study. 106 patients were enrolled in the coronary rehabilitation group and 140 patients in the noncoronary rehabilitation group. The demographical characteristics and clinical data of the two groups are shown in Table 1. In the demographical part, it showed that the patients in the coronary rehabilitation group were younger than those in the noncoronary rehabilitation group, and the results were statistically significant (*P*=0.001), and the BMI of the coronary rehabilitation group was lower than that of the noncoronary rehabilitation group (*P*=0.003). There were also significant differences in the time between the most recent MI (*P*=0.011) and the percutaneous coronary intervention type in the same period (*P*=0.001). As for follow-up treatment, more patients in the coronary rehabilitation group received drug-eluting stent treatment (*P*=0.007). In terms of comorbidities, the coronary rehabilitation group had a higher proportion of heart failure (*P*=0.004) and hypertension (*P*=0.015). There were no significant differences on gender and smoking status (*P* > 0.05). There were no statistical differences in the proportion of diabetes, chronic lung disease, cerebrovascular disease, and tumor (*P* > 0.05). After the propensity match, there were no statistical differences in the variables listed in Table 2 (all *P* > 0.05).

### 3.2. Primary Endpoint

During the average (38.9 ± 22.5) months of follow-up, there were 37 primary endpoint events (all-cause deaths), including 28 cardiovascular deaths and 9 noncardiovascular deaths. As shown in Table 3, the hazard ratio (HR) of coronary rehabilitation for primary endpoint was 0.465 95% CI (0.233–0.926) (*P*=0.029). Survival analysis also showed that the survival rate of the coronary rehabilitation group was higher than that of the noncoronary rehabilitation group (*P*=0.024).

### 3.3. Secondary Endpoint

During the follow-up period, 44 secondary endpoint events occurred, including 18 cases of myocardial infarction and 26 cases of emergency revascularization. Compared with the noncoronary rehabilitation group, the risk of cardiac events in the coronary rehabilitation group was significantly lower, with HR of 0.532 95% CI (0.287–0.984) (*P*=0.044). There were no statistical significance in subgroup analysis of myocardial infarction and emergency revascularization (*P* > 0.05). The Kaplan–Meier survival curve showed that the coronary rehabilitation group had fewer cardiovascular events than the noncoronary rehabilitation group (*O* = 0.039).

## 4. Discussion

As far as we know, this study retrospectively compared patients treated with coronary rehabilitation and patients who did not receive coronary rehabilitation. It was the first time that coronary rehabilitation can effectively reduce all-cause mortality and cardiac events in patients with CKD after percutaneous coronary intervention. It is worth mentioning that, in this study, the conclusions were more convincing as baseline bias was eliminated by propensity score matching.

Previous studies had provided a close link between coronary rehabilitation training and the reduction of all-cause mortality [15]. A systematic review and meta-analysis of 148 randomized controlled trials with a total of 97,486 participants strengthened the reduction of mortality in people with coronary heart disease through coronary rehabilitation [16]. However, there are still some controversies regarding the indications and risks of coronary rehabilitation, especially for high-risk patients. Some studies had found that coronary rehabilitation was less effective in diabetic patients [17, 18], and one study found that coronary rehabilitation had the same effect in DM patients as in non-DM patients [19]. Those controversies required more researches to focus on specific patients, especially patients with some complications.

CKD is an independent risk factor for CAD. CAD is the main cause of incidence rate and mortality of CKD patients [20–22]. For patients undergoing percutaneous coronary intervention, even in the era of drug-eluting stents, CKD complications can lead to higher surgical complications, restenosis, and future cardiac events [23]. Compared with patients of simple CKD or CAD, patients with both CKD and CAD have a higher risk of death and cardiac events. Some studies have investigated the effectiveness of coronary rehabilitation for CAD patients, which suggested that coronary rehabilitation can significantly improve renal function and reduce the coronary artery risk in CKD patients [24–27]. However, no previous studies have observed the long-term effects of coronary rehabilitation on CKD patients. Propensity score matching eliminates baseline features that may affect survival, including age, BMI, the percutaneous coronary intervention emergency, most recent mitral insufficiency (MI) history, cardiac function, and other complications. After the propensity match, there was no statistical significance.

Univariate Cox regression analysis was performed between the two groups to compare the all-cause and mortality and cardiac events in the coronary rehabilitation group and the noncoronary rehabilitation group. The result was positive which was caused by two main mechanisms. On the one hand, coronary rehabilitation complexes including exercise, smoking cessation, and weight loss have been shown to be beneficial to endothelial function, which may play a role in improving renal function and revascularization of coronary arteries [28]. On the other hand, some studies have showed that coronary rehabilitation can reduce the level of oxidized low-density lipoprotein (ox-LDL), which is essential for the development and deterioration of CAD [29].

No matter how great the benefits of coronary rehabilitation are, without people participation and compliance, the result is nonsense. Despite years of promotion, the participation rate of coronary rehabilitation is still very low, especially in countries with undeveloped medical conditions. According to the Canadian Institutes of Health Research, only 38.8% of countries have heart rehabilitation programs, of which 68.0% are in high income countries and 23% are in low and middle income countries [12]. In China, a survey showed that only 30 out of 124 people (24%) said they had initiated the coronary rehabilitation program [30]. The main obstacles hindering the coronary rehabilitation program are low referral rate, poor patient compliance, lack of doctor approval, obesity, multiple diseases, poor or no exercise habits, smoking, mental health, traffic problems, lack of social support, and lack of rest time [31]. In this study, approximately 46% (106 out of 246) CKD patients participated in the coronary rehabilitation program, which is above average, which could be attributed to the complete coronary rehabilitation team.

It should also be noted that there are several limitations of this study. Firstly, retrospective design has effect on the strength of evidence. Secondly, the follow-up data are not as good as the cohort study, the proportion of censored data is relatively high, and there may be a certain deviation in the final result. Finally, because the clinical data of CKD are incomplete, this study lacked CKD staging information.

## 5. Conclusions

In conclusion, this study demonstrated that long-term coronary rehabilitation program would effectively reduce the risk of death and the incidence of cardiac events in patients with CKD. More efforts are needed to promote coronary rehabilitation in patients with CAD, especially for those with CKD.

## Figures and Tables

**Table 1:** Demographical characteristics and clinical data of the coronary rehabilitation group and the noncoronary rehabilitation group before propensity score match.

Variables	The coronary rehabilitation group (*n* = 106)	The noncoronary rehabilitation group (*n* = 140)	*P* value
Demographics			
Age (y, mean ± SD)	58.4 ± 17.5	65.7 ± 17.2	0.001
Gender (male %)	65 (61.3%)	76 (54.3%)	0.299
BMI (kg/m^−2^)	22.8 ± 3.1	24.0 ± 3.2	0.003
Smoking (%)	37 (34.9%)	48 (34.3%)	1.000
Most recent MI			0.011
<24 h	24 (22.6%)	54 (38.6%)	
1–7 d	17 (16.0%)	19 (13.6%)	
>7 d	25 (23.6%)	15 (10.7%)	
Never	40 (37.7%)	52 (37.1%)	
Unstable angina	76 (71.7%)	92 (65.7%)	0.336
Prior percutaneous coronary intervention	16 (15.1%)	32 (22.9%)	0.145
Prior CABG	13 (12.3%)	25 (17.9%)	0.286
Contemporary percutaneous coronary intervention			0.001
Emergency percutaneous coronary intervention	23 (21.7%)	51 (36.4%)	
Urgent percutaneous coronary intervention	43 (40.6%)	65 (46.4%)	
Elective percutaneous coronary intervention	40 (37.7%)	24 (17.1%)	
Drug-eluting stent	48 (45.3%)	39 (27.9%)	0.007
GP IIb/IIIa use	66 (62.3%)	76 (54.3%)	0.241
LVEF	49.1 ± 12.2	53.3 ± 11.4	0.006
Comorbidities			
Heart failure	31 (29.2%)	19 (13.6%)	0.004
Hypertension	66(62.3%)	65 (46.4%)	0.015
Diabetes mellitus	22 (20.8%)	27 (19.3%)	0.872
Chronic lung disease	26 (24.5%)	31 (22.1%)	0.760
Cerebrovascular disease	1 (0.9%)	6 (4.3%)	0.244
Tumor	8 (7.5%)	5 (3.6%)	0.249

BMI, body mass index; MI, myocardial infarction; CABG, coronary artery bypass graft; LVEF, left ventricular ejection fraction.

**Table 2:** Demographical characteristics and clinical data of the coronary rehabilitation group and the noncoronary rehabilitation group after propensity score match.

Variables	The coronary rehabilitation group (*n* = 89)	The noncoronary rehabilitation group (*n* = 89)	*P* value
Demographics			
Age (y, mean ± SD)	59.9 ± 17.7	61.3 ± 17.8	0.517
Gender (male %)	59 (66.3%)	64 (71.9%)	0.219
BMI (kg/m^−2^)	23.1 ± 3.0	23.5 ± 3.1	0.406
Smoking(%)	29 (32.6%)	27 (30.3%)	0.872
Most recent MI			0.503
<24 h	24 (27.0%)	30 (33.7%)	
1–7 d	17 (19.1%)	15 (16.9%)	
>7 d	15 (16.9%)	9 (10.1%)	
Never	33 (37.1%)	35 (39.3%)	
Unstable angina	61 (68.5%)	56 (62.9%)	0.528
Prior percutaneous coronary intervention	12 (13.5%)	14 (15.7%)	0.832
Prior CABG	11(6.7%)	19 (21.3%)	0.160
Contemporary percutaneous coronary intervention			0.301
Emergency percutaneous coronary intervention	23 (25.6%)	30(33.7%)	
Urgent percutaneous coronary intervention	33 (37.1%)	35 (39.3%)	
Elective percutaneous coronary intervention	33 (37.1%)	24 (27.0%)	
Drug-eluting stent	34 (38.2%)	28 (31.5%)	0.432
GP IIb/IIIa use	51 (57.3%)	52 (58.4%)	1.000
LVEF	49.8 ± 12.3	51.9 ± 12.4	0.243
Comorbidities			
Heart failure	24 (27.0%)	19 (21.3%)	0.484
Hypertension	50(56.2%)	42 (47.2%)	0.294
Diabetes mellitus	19 (21.3%)	18 (20.2%)	1.000
Chronic lung disease	15 (16.9%)	10 (11.2%)	0.389
Cerebrovascular disease	1 (1.1%)	5 (5.6%)	0.211
Tumor	1 (1.1%)	2 (2.2%)	1.000

BMI, body mass index; MI, myocardial infarction; CABG, coronary artery bypass graft; GP, glycoprotein; LVEF, left ventricular ejection fraction.

**Table 3:** Hazard ratio (HR) of endpoint for patients treated with coronary rehabilitation compared with patients without coronary rehabilitation.

	HR	95% CI	*P* value
Primary endpoint	0.465	0.233–0.926	0.029
Secondary endpoint			
Myocardial infarction	0.465	0.174–1.239	0.125
Emergent revascularization	0.482	0.264–1.285	0.180
Overall	0.532	0.287–0.984	0.044

## Data Availability

The data that support the findings of this study are available from the corresponding author upon reasonable request.
